RETRACTED

# Pattern and In-Hospital Mortality of Thoracoabdominal Injuries Associated with Motor Vehicle Accident-Related Spinal Injury: A Retrospective Single-Center Study

**DOI:** 10.1155/2021/9514169

**Published:** 2021-10-21

**Authors:** Mubarak Ali Algahtany, Walid Abd El Maksoud

**Affiliations:** ^1^Division of Neurosurgery, Department of Surgery, College of Medicine, King Khalid University, Abha, Saudi Arabia; ^2^Division of General Surgery, Department of Surgery, College of Medicine, King Khalid University, Abha, Saudi Arabia

## Abstract

**Background:**

Motor vehicle accident (MVA) is a global health hazard that results in spinal, thoracic, and abdominal injuries. Detailed studies on the association between MVA-related traumatic spinal injury (TSI) and thoracoabdominal injuries are lacking. This study aims to elucidate the prevalence, pattern of association between these injuries, and related outcomes in terms of in-hospital mortality.

**Methods:**

This is a retrospective single-center study of MVA-related TSI with thoracoabdominal associated injuries. Descriptive analysis was performed for gender, age, spinal injury level, thoracoabdominal injury region, admission day, hospital stay duration, and discharge category. The association between TSI and thoracoabdominal injury was analyzed, and the chi-square test was used to test the significance of differences. A statistically significant difference was considered at *P* values less than 0.05.

**Results:**

The cohort had a mean age of 33.6 ± 17.7 years with predominantly more males (85.1%). Thoracoabdominal injuries were present in 10.5% of MVA-related TSIs, and 9.2% of victims died during their hospital stay. There is a significant (*P*=0.045) association between the level of the spinal and the region of thoracoabdominal injuries. The presence of TSI-associated thoracic injury significantly (*P*=0.041) correlated with increased in-hospital mortality more than abdominal injury.

**Conclusion:**

Thoracoabdominal injuries concomitant with MVA-related TSI cause considerable mortality. A pattern of association exists between the level of spinal and region of thoracoabdominal injury. Knowledge of this pattern is helpful in the routine practice of trauma health partitioners.

## 1. Introduction

Traumatic spinal injury (TSI) is an infrequent trauma-related injury yet having a considerable risk for causing permanent disability and death [1]. Worldwide, motor vehicle accident (MVA) is the principal reason for TSI, causing between 21% and 34% of all TSIs, while accounting for 80% of TSIs in Saudi Arabia [2–4].

Moreover, MVA usually results in polytrauma depending on gender, age, speed of the vehicle, and type of accident [5, 6]. Of these multiple injuries, thoracic and abdominal traumas are common [7, 8]. Thoracic ranks second to head injury in the number of fatalities and serious injuries, while abdominal injury accounts for 10% of trauma-related deaths following MVAs [9, 10].

RETRACTED

Traumatic spinal injuries, though less frequent, can cause debilitating consequences and often are accompanied by other organ injuries such as the head, chest, abdomen, and extremity [11]. The coexistence of trauma-related injuries is well known, yet few studies investigated the association between TSI and thoracoabdominal injuries and the related clinical outcomes [12]. The association between the spinal and thoracoabdominal injuries, however, is suggested by the anatomical proximity between the thoracic spine and the thoracic cage, as well as between the lumbar spine and abdominal viscera. The incidence of this association is higher following MVA due to its high potential for multiorgan injuries [1, 2, 12]. Furthermore, since polytrauma patients are initially seen in urgent circumstances, the apparent injury may attract the most attention, risking overlooking occult associated injuries [13]. The in-depth analysis of the pattern of associations between MVA-related injuries is valuable to predict and attend concomitant injuries, hence improve outcome and reduce under or over triage [8].

This study aims to provide this information and determine the incidence, pattern, and in-hospital mortality of thoracoabdominal injuries coexisting with spinal injuries due to motor vehicle accidents.

### 1.1. Patients and Methods

The study followed a retrospective design. All injured patients admitted from January 2010 to January 2020 to Aseer Central Hospital, which is the main tertiary hospital in southern Saudi Arabia, were revised.

The inclusion criteria comprised all patients who were 14 years old or more, admitted due to MVA and had a documented spinal injury in addition to thoracic and/or abdominal injuries. Patients with spinal injuries due to other causes and patients without simultaneous thoracic nor abdominal injuries were excluded from the study.

The files of the studied patients were reviewed for date of admission, demographic data, details of the spinal injuries, details of the thoracic and/or abdominal injuries, duration of hospital stay, the need of critical care admission, and prognosis on discharge.

### 1.2. Outcomes

The primary endpoints were as follows:

- Determination of the incidence of MVA-related TSIs associated with thoracoabdominal injuries
- Determination of the pattern of thoracoabdominal injuries that are associated with MVA-related TSI
- Determination of the in-hospital outcome of MVA-related TSIs associated with thoracoabdominal injuries

RETRACTED

### 1.3. Statistical Analysis

The statistical analysis of data was performed using the Statistical Package for Social Sciences (SPSS version 25; SPSS Inc., Chicago, Illinois, USA). Descriptive statistics were applied (i.e., frequency and percentage for categorical data in addition to mean and standard deviation for quantitative data). The chi-square likelihood ratio was used to test the significance of differences. A statistically significant difference was considered at *P* values less than 0.05.

The research was approved by the ethical committee of King Khalid University (ECM#2021-4001). All precautions were taken to conceal the identity of the patients.

## 2. Results

Out of the 827 patients admitted with MVA-related spinal injuries during the study period, 87 patients (10.5%) had associated thoracic and/or abdominal injuries. The age of the studied group ranged from 14 to 87 years with a mean of 33.6 ± 17.7 years, and the majority (57.5%) were aging between 20 and 40 years. The study included 74 males (85.1%) and 13 females (14.9%). Spinal injuries were coupled with chest injuries in 58 patients (66.7%), abdominal injuries in 22 patients (25.3%), and both thoracic and abdominal injuries in 7 patients (8.0%). Demographic and clinical data of the studied group are shown in Table 1.

Regarding the anatomical site of the spinal injury, thoracic (32.2%) followed by the cervical spine (26.4%) were the most affected spinal levels (Table 1). We found a significant association between the region of thoracoabdominal injury and the level of the spinal injury (*P* = 0.045) (Table 2). The associated thoracic injury was more prevalent in patients with cervical and dorsal spine injures, while the concomitant abdominal injury was more common in patients with sacral and lumbar spine injures.

Regarding the type of thoracoabdominal injuries associated with MVA-related TSI, rib fractures (46.6%) and lung contusions (25.9%) were the commonest types of thoracic injures (Table 3). At the same time, splenic (59.1%) and liver injuries (18.2%) were the most common abdominal injuries.

Significantly more patients were admitted during weekdays than weekends (*P* = 0.014) (Table 4). The in-hospital mortality was 9.2%. In addition, all patients who expired had thoracic injuries (*P* = 0.041). There were no differences between thoracic and abdominal injuries in terms of day of admission (weekdays vs. weekends), hospital stay duration, need for intensive care, or prevalence of traumatic spinal cord injury.

## 3. Discussion

Motor vehicles are the primary transportation method in Saudi Arabia, leading to many MVA-related injuries and mortalities over the past two decades [14, 15]. It is estimated that MVAs cause four injuries hourly and nineteen deaths daily in the country [16]. Motor vehicle accidents are also a global issue that causes nearly half of the trauma-related deaths in the USA [7].

RETRACTED

The motor vehicle accident is a high-energy trauma mechanism with substantial risk for multiple spinal and nonspinal injuries [17]. The odd for MVA-related multiple injuries increases with the vehicle speed at the collision [8, 9]. Among MVA-related injuries, thoracoabdominal injuries are serious. Around one-tenth and one-fourth of MVA-related deaths are attributed to abdominal and thoracic injuries, respectively [7, 10]. Furthermore, the risk of spinal injuries increases in the presence of thoracic and abdominal injuries [18].

Though traumatic spinal injury accounts only for 10% of trauma-related admissions, it has a considerable threat to cause death and permanent disability [1, 19, 20]. Additionally, polytrauma victims with TSI have less satisfactory outcomes than those with no spinal injury [20].

The mortality from TSI has not changed over the last two decades [18]. A thorough analysis of the reasons behind this nonchanging mortality trend has not been done. The presence of associated injuries is a plausible contributing factor for several reasons. Firstly, coexistent nonspinal injuries are present in over half of the TSI patients [21–23]. Secondly, the presence of TSI increases the odd of concomitant thoracoabdominal injuries by several folds [20, 24]. Finally, the coexistence of TSI and other nonspinal accompanying injuries has been shown to increase mortality [2].

The detailed analysis of the association mentioned above is more crucial following traffic accidents because MVA is the leading cause for TSI and results in more TSI-associated other injuries than a lower energy mechanism such as fall [2, 19, 22, 23]. This comprehensive analysis will allow better disease understanding and more effective injury prevention. In this context, this study aimed to provide detailed information on the association between TSI and thoracoabdominal injuries following MVAs.

We found more male victims of MVA-related TSI with thoracoabdominal associated injuries than females. This is consistent with most studies on MVA-related TSI [25]. The very high male percentage reported here is coherent with other studies from Saudi Arabia [21, 26]. The explanation is likely cultural and legislative factors, including a previous pan on women driving, rather than anatomical or physiological factors [15].

Patients in the 20–40 years age group were the most affected in our study. This is similar to results from local and regional studies on MVA-related TSI [2, 21]. Globally, the mean age of TSI is 40 years, with a tendency to increase in developed countries while decreasing in low-income nations [19].

RETRACTED

Most patients were admitted on weekdays than weekends which is likely related to using motor vehicles as the primary mechanism of transport to work.

The thoracic spine was the most affected level in our study (32.2%), followed by the cervical spine (26.4%). This is close to the finding of 28.06% thoracic and 24.50% cervical involvement from one sizeable European study [18]. The level of spinal involvement, however, is variable between studies largely due to the study population and inclusion criteria [12, 23, 27]. The main explanation for the distribution we have seen in this study could be limiting TSIs to those with concomitant thoracoabdominal injuries exclusively due to MVA. Therefore, the predominance of thoracic spine injury in this cohort is attributed to the 67% ratio of chest injury among the study group. Furthermore, the cervical and thoracic spinal levels are common locations for TSI following MVA [22].

Chest injury was 2.6 times more common than abdominal injury in this study. This is in liaison with reports stating thoracic injury as one of the commonest MVA-related injuries [7, 9]. Thoracic trauma commonly accompanies TSIs, especially at the dorsal spinal level. One study found thoracic injury in 41% of TSI patients, ranking as the commonest TSI-associated injury [23]. Another study found increased odds of pulmonary injury by multiple folds in the presence of thoracic spinal trauma [24].

Our finding of fewer abdominal than thoracic injury coexisting with TSI is coherent with others [18]. Abdominal injury, however, still commonly coexists with TSI, and studies have found abdominal injury odd to increase three folds in the presence of thoracic spine and five folds in association with lumbar spine injuries [20, 24]. This association is more obvious following MVA, with one report stating associated intra-abdominal injuries among 10% of lumbar spine injuries with 73% of those due to MVA [28].

Combined thoracic and abdominal injuries were uncommon (8%) in this cohort. This could be related to the complex interaction between the vehicle, its occupant, and the collision nature. The car roll-over mechanism increases the risk for multiple TSI-associated injures by several folds [2]. In frontal impacts, restrained front seat occupants tend to receive injuries from the steering wheel to the chest [29, 30], while car occupants with forwarding flexion mechanisms had injuries to the lumbar spine, with primarily concurrent abdominal injuries [27].

RETRACTED

The introduction of the seat belt led to a complex pattern of thoracoabdominal injuries, which are more common in the presence of thoracolumbar spine injury [31]. Thoracic injuries due to seat belt force include sternal fracture, rib fracture, pulmonary contusion, and myocardial contusion [32]. In agreement with that, rib fracture constituted the major associated injury in our study, representing 46.6% of the chest injuries and 31.0% of the total concomitant injuries.

Splenic and liver injuries were the most common abdominal injuries in our study. This could be related to the lower ribs' fractures and physical forces transmission around the seat belt point of contact [8].

The mortality in this group was 9.2% which is at the upper end of the reported range of TSI mortality [1, 19]. This indicates that the presence of TSI-associated thoracoabdominal injuries is a predictor of increased mortality. Specifically, all fatalities in this study had combined thoracic spine and chest injuries. The increased mortality of TSI patients suffering concomitant thoracic compared to abdominal injuries appears to be an inherent problem linked to thoracic trauma rather than increased injury severity. This is supported by the lack of differences between the two sites of injury in terms of day of admission (weekdays vs. weekends), hospital stay duration, need for intensive care, or prevalence of traumatic spinal cord injury. This is consistent with the literature indicating that thoracic spine injury and chest injury are predictors of increased mortality and poorer outcomes [18, 20, 26].

### 3.1. Limitation

This study is limited by its retrospective and hospital-based nature. It also lacked accident details and assessment of injury severity by validated scales like injury severity score. Nonetheless, it provides new data pertinent to a global major health hazard of MVA-related injuries. Furthermore, the results from this study are relevant to the daily practice of healthcare providers caring for trauma patients.

## 4. Conclusion

Concurrent thoracoabdominal injuries are present in one-tenth of MVA-related TSIs and generate significant mortality risk. A pattern of association exists between the spinal injury level and thoracoabdominal injury type, impacting the in-hospital outcomes. Thorough knowledge of this pattern is valuable to prevent overlooking TSI-associated occult injuries and improving outcomes.

## Figures and Tables

**Table 1:** Demographics and outcome of motor vehicle accident-related traumatic spinal injuries associated with thoracoabdominal injuries (*n* = 87).

	No.	%
Age		
<20 years	16	18.4
20–40 years	50	57.5
>40 years	21	24.1
*Gender*		
Males	74	85.1
Females	13	14.9
*Day of admission*		
Weekday	58	66.7
Weekend	29	33.3
*Thoracoabdominal associated injury*		
Chest	58	66.7
Abdomen	22	25.3
Both	7	8.0
*Nonthoracoabdominal associated injuries*	49	56.3
*Level of spinal injury*		
Cervical	23	26.4
Thoracic	28	32.2
Lumber	14	16.1
Sacral	10	11.5
Multiple levels	12	13.8
*Hospital stay*		
<10 days	28	32.2
10–20 days	27	31.0
>20 days	32	36.8
*Discharge category*		
Expired	8	9.2
Home	77	88.5
Transferred	2	2.3
*Admission to intensive care unit*		
No	76	87.4
Yes	11	12.6
*Traumatic spinal cord injury*		
No	78	89.7
Yes	9	10.3

RETRACTED

**Table 2:** Association between thoracoabdominal injuries and level of the spinal injury (*n* = 87).

Level of spinal injury	Thoracic injury (*n* = 58)		Abdominal injury (*n* = 22)		Both (*n* = 7)		Total (*n* = 87)		*P* value^†^
	No.	%	No.	%	No.	%	No.	%	
Cervical	18	31.0	3	13.6	2	28.6	23	26.4	0.045^*∗*^
Thoracic	22	37.9	3	13.6	3	42.9	28	32.2	
Lumbar	8	13.8	5	22.7	1	14.3	14	16.1	
Sacral	3	5.2	6	27.3	1	14.3	10	11.5	
Multiple levels	7	12.1	5	22.7	0	0.0	12	13.8	

^†^Based on the likelihood-ratio chi-square statistic. ^*∗*^*P* < 0.05 is significant.

**Table 3:** Breakdown of thoracoabdominal injuries associated with motor vehicle accident-related traumatic spinal injuries.

Injuries^*∗*^	Thoracic	Abdominal	Both	Total
	No. (%)	No. (%)	No. (%)	No. (%)
Unspecified chest injury	6 (10.3)	0 (0.0)	1 (14.3)	7 (8.0)
Fracture ribs	23 (39.6)	0 (0.0)	4 (57.1)	27 (31.0)
Fracture sternum	6 (10.3)	0 (0.0)	0 (0.0)	6 (6.8)
Hemopneumothorax	3 (5.2)	0 (0.0)	0 (0.0)	3 (3.4)
Hemothorax	6 (10.3)	0 (0.0)	0 (0.0)	6 (6.8)
Pneumothorax	11 (18.9)	0 (0.0)	0 (0.0)	11 (12.6)
Lung contusion	13 (22.3)	0 (0.0)	2 (28.6)	12 (13.8)
Open wound of thorax	1 (1.7)	0 (0.0)	0 (0.0)	1 (1.1)
Unspecified abdominal injury	0 (0.0)	8 (36.4)	2 (28.6)	10 (11.5)
Liver injury	0 (0.0)	3 (13.6)	1 (14.3)	4 (4.6)
Spleen injury	0 (0.0)	9 (40.9)	4 (57.1)	13 (14.9)
Kidney injury	0 (0.0)	1 (4.5)	0 (0.0)	1 (1.1)
Injury of urinary bladder	0 (0.0)	1 (1.7)	0 (0.0)	1 (1.1)
Rectal injury	0 (0.0)	1 (4.5)	0 (0.0)	1 (1.1)
Anal tear	0 (0.0)	2 (9.1)	0 (0.0)	2 (2.3)

^*∗*^Coexistence of several injuries occurred in some patients.

**Table 4:** Association between the different variables and thoracoabdominal injuries associated with motor vehicle accident-related traumatic spinal injuries (*n* = 87).

Variables	Thoracic injury (*n* = 58)		Abdominal injury (*n* = 22)		Both (*n* = 7)		Total (*n* = 87)		*P* value^†^
	No.	%	No.	%	No.	%	No.	%	
*Age*									
<20 years	7	43.8	8	50.0	1	6.3	16	18.4	0.065
20–40 years	33	66.0	12	24.0	5	10.0	50	57.5	
>40 years	18	85.7	2	9.5	1	4.8	21	24.1	
*Gender*									
Males	51	68.9	18	24.3	5	6.8	74	85.1	0.492
Females	7	53.8	4	30.8	2	15.4	13	14.9	
*Day of admission*									
Weekday	34	58.6	17	29.3	7	12.1	58	66.7	0.014^*∗*^
Weekend	24	82.8	5	17.2	0	0.0	29	33.3	
*Hospital stay*									
<10 days	16	27.6	10	45.5	2	28.6	28	32.2	0.488
10–20 days	21	36.2	4	18.2	2	28.6	27	31.0	
>20 days	21	36.2	8	36.4	3	42.9	32	36.8	
*Discharge category*									
Expired	8	13.8	0	0.0	0	0.0	8	9.2	0.041^*∗*^
Home	49	84.5	22	0.0	6	85.7	77	88.5	
Transferred	1	1.7	0	0.0	1	14.3	2	2.3	
*Admission to intensive care unit*									
No	49	64.5	20	26.3	7	9.2	76	87.4	0.580
Yes	9	81.8	2	18.2	0	0.0	11	12.6	
*Traumatic spinal cord injury*									
No	52	66.7	19	24.4	7	9.0	78	89.7	0.802
Yes:	6	66.7	3	33.3	0	0.0	9	10.3	

^†^Based on the likelihood-ratio chi-square statistic. ^*∗*^*P* < 0.05 is significant.

RETRACTED

## Data Availability

The data used in this study are available from the corresponding author upon request.
